# Development of a Pressure-Sensitive Conductive Rubber Sensor for Analyzing Meniscal Injury in Porcine Models

**DOI:** 10.1155/2021/4931092

**Published:** 2021-11-03

**Authors:** Shunsuke Sezaki, Shuhei Otsuki, Kuniaki Ikeda, Nobuhiro Okuno, Yoshinori Okamoto, Hitoshi Wakama, Tomohiro Okayoshi, Masashi Neo

**Affiliations:** ^1^Department of Orthopedic Surgery, Osaka Medical and Pharmaceutical University, 2-7 Daigakumachi Takatsuki, Osaka 569-8686, Japan; ^2^QOL Research Laboratory, Gunze Limited, 1 Zeze Aonotyo Ayabe, Kyoto 623-8511, Japan

## Abstract

The assessment of the distribution of contact pressure on the meniscus is important in the elucidation of kinematics, etiology of joint diseases, and establishment of treatment methods. Compared with sensors widely used in recent years, pressure-sensitive conductive rubber sensors are easy to mold, flexible, durable, and resistant to shearing forces. This study is aimed at developing a rubber sensor for meniscal research and evaluating the pressure distribution after meniscal injury using porcine models. After confirming the reliability of the rubber sensor, contact pressure was obtained from the rubber sensor using the medial meniscus and femur of the porcine knee. Three test conditions of intact meniscus, radial tear, and meniscectomy were prepared, and a compressive load of 100 N was applied. After confirming the high reliability of the rubber sensor, the intact meniscus had the most uniform pressure distribution map, while the pressure in the meniscectomy model was concentrated in the resection region. The high-pressure region was significantly smaller in the intact group than in the radial tear models after 80 and 100 N (*P* < 0.05). The rubber sensor captured the pressure concentration specific to each examination group and was useful for evaluating the relationship between the pattern of meniscal injury and changes in the biomechanical condition of the knee.

## 1. Introduction

The role of the meniscus in load transmission and shock absorption is widely recognized [1–4]. Meniscal damage and partial or total meniscectomy following injury have been shown to dramatically increase the contact stress on the articular surface [5–8].

The assessment of the distribution of contact pressure in the menisci is important for elucidating the kinematics and the etiology and treatment of joint diseases. Recently, the Tekscan pressure-sensitive film sensor (Tekscan Inc., Boston, MA, USA) [3, 9–11] or a pressure-sensitive paper (Prescale, Fuji Film, Tokyo, Japan) [12–14] has been widely used to measure the contact pressure in human or large-animal knee joint, and thus, the function of menisci has been clarified. However, these sensors are unsuitable for use in areas where shear forces are applied, and use in heavily deformed contact surfaces causes wrinkling of the film. Moreover, it is difficult to evaluate pressure-sensitive paper because the pressure distribution is represented by gradients of a single color, and it is necessary to replace the sensor for each test [15].

Therefore, we focused on a pressure-sensitive conductive rubber sensor because it is easy to mold, flexible, and durable and can be used to evaluate shear forces [16]. This device is a sensor that converts the amount of rubber displacement into pressure [17] and has already demonstrated reliability in robotics, medical devices, and body pressure distribution measurements. However, the use of a sensor with rubber has not been reported in the biomechanical analysis of menisci or tibiofemoral contact pressure.

We hypothesized that meniscal research using this novel sensor would provide a new method for functional and biomechanical analyses.

This study is aimed at developing a novel pressure-sensitive conductive rubber sensor and evaluating the pressure dispersion after meniscal injury in porcine models.

## 2. Materials and Methods

### 2.1. Novel Pressure-Sensitive Conductive Rubber Sensor

A pressure-sensitive conductive rubber sensor was developed to improvise the Inastomer sensor (Inaba Rubber Co., Ltd., Osaka, Japan). The sensor was established with a base of 20 mm, a sensor pitch of 1 mm, 400 sensing points, and a thickness of 0.8 mm (Figure 1). Before examination, calibration was performed at 5 MPa using calibration equipment dedicated to this system. The results were calculated for this device to the second decimal place. The color map can be obtained by the commercial software.

### 2.2. Reliability of the Novel Pressure-Sensitive Conductive Rubber Sensor

Pressures equivalent to 0.1, 0.2, 0.3, 0.5, 1.0, and 2.0 MPa were applied to the pressure sensor by a universal testing machine (Autograph AGS-X, Shimadzu Corporation, Kyoto, Japan) with a *φ*10 mm jig (Figure 2). The test was performed at least three times at each pressure. The compressive force applied by the universal testing machine and the mean pressure calculated from the device were compared. The intraclass correlation coefficient (ICC) of intraobserver reliability was calculated using the pressure calculated from the device to demonstrate the reliability of its evaluation.

### 2.3. Pressure Conditions and Measurement of Distribution

Five fresh porcine knees of 6 months of age were used in this study. The femur and medial meniscus were marked for alignment at the full extension position, and they were removed. The average medial meniscal size was 30 mm in length and 15 mm in width. To perform a compression test using a universal test machine, the femur was fixed to a special jig that can be tightened in six places with screws. Two holes for screw insertion were made in the anterior-posterior direction of the femur, and screws were inserted into the holes. After adjusting the femur to be horizontal, the surroundings were fixed with the remaining four screws. The meniscus was fixed to a flat synthetic bone and set according to the marked alignment (Figure 3(a)). During the load test, we visually confirmed that it could fit the artificial bone and was not unstable, and then, we conducted the experiment. A pressure sensor was inserted between the meniscus and the flat synthetic bone, and a compression test was performed at a speed of 25 N/s, a maximum load of 100 N, and 60 s after reaching 100 N [14]. The mean contact pressure and contact area were calculated using the pressure sensor after reaching 100 N. Furthermore, the contact area was calculated every 20 N, and an area over 0.4 MPa was defined as high pressure. Regarding the placement of the color map, a photograph, including the meniscus and the sensor, was taken prior to the test, and the color map was placed on the meniscus by synthesizing the position of the sensor and the color map.

### 2.4. Meniscal Injury Models

Using scalpel #11, meniscal injury models were created to simulate commonly seen meniscal damage [14]. The morphology of the created lesions was a radial tear involving 90% of the body width and partial meniscectomy involving 60% of the central meniscus. All knees were tested under three conditions: (1) intact (Figure 3(b)), (2) radial tear extending 90% (Figure 3(c)), and (3) meniscectomy of the central 60% (Figure 3(d)).

### 2.5. Statistical Analysis

All data analyses were performed using JMP Pro version 15 (SAS Institute Japan Ltd., Tokyo, Japan). The calculated data were expressed as average values ± standard deviation. Dunn's multiple comparison method was used to analyze the differences between groups. Statistical significance was set at *P* < 0.05.

## 3. Results

The calculated pressures from the sensor were 0.13 ± 0.02, 0.21 ± 0.02, 0.28 ± 0.02, 0.43 ± 0.04, 0.98 ± 0.05, and 2.01 ± 0.34 MPa, which correlated with the applied pressure from 0.1 to 2.0 MPa, respectively, and the ICC was 0.96 (Figure 4(a)). Color maps for each pressure are shown in Figure 4(b).

A representative distribution map of each model obtained from the rubber sensor is shown in Figures 5(a)–5(c). The mean contact pressure in meniscectomy (0.31 ± 0.05 MPa) was significantly larger than that in intact (0.21 ± 0.03 MPa) and radial tear (0.23 ± 0.01 MPa) (*P* < 0.05, Figure 5(d)). The peak contact pressure of the intact was the smallest (0.43 ± 0.02 MPa), and the meniscectomy was the largest (1.04 ± 0.19 MPa), with a significant difference in all groups (*P* < 0.05, Figure 5(e)). The mean contact area in meniscectomy (60.00 ± 1.73 mm^2^) was significantly smaller than that in intact (99.67 ± 13.05 mm^2^) and radial tear (111.33 ± 7.77 mm^2^) (*P* < 0.05, Figure 5(f)).

Regarding the contact area analyzed every 20 N, there was no area above 0.5 MPa in intact. In contrast, high-pressure areas, over 0.4 MPa, were significantly larger in radial tear and meniscectomy than in intact when a load of 80 and 100 N was applied (*P* < 0.05, Figure 6(a)). The pressure distribution showed that the most uniform map was obtained in intact, whereas high-pressure regions were detected around the radial tear and meniscectomy conditions (Figure 6(b)).

## 4. Discussion

The most important finding of this study is that the novel pressure-sensitive conductive rubber sensor is a reliable device that is appropriate for evaluating the pressure distribution of meniscal injuries in porcine models.

The Tekscan sensor has been widely used for the biomechanical analysis of the knee joint because of its accuracy and reliability. In contrast, it has been reported to have a shorter life under harsh load conditions [15], indicating that it might not be cost-effective. We focused on a pressure-sensitive conductive rubber sensor because it is thin and has excellent flexibility [16]. Furthermore, this sensor can endure harsh stress conditions in several fields, indicating that cost-effectiveness might be another attractive feature for its use in biomechanical studies. The rubber sensor shows not only cost-effectiveness but also appropriate accuracy and reliability in the present *in vitro* study. Moreover, this sensor can be mounted on curved surfaces, which is an added advantage of rubber sensors [16]. This property indicates that better accuracy in pressure distribution was obtained even on complex geometric surfaces within the knee joint.

In the next stage, three conditions (intact, radial tear, and partial meniscectomy) were evaluated using porcine knees. Intact menisci showed the most uniform pressure distribution with respect to the hoop function. In addition, the results of the radial tear model were similar to those of previous reports [9] that radial tear had significantly higher maximum pressures with smaller contact areas than intact. In the current study, there was a significant difference in high-pressure distribution and degree among the meniscal injury models. Importantly, the radial tear model showed the high-pressure area to be locally concentrated around the tear. It was suggested that the damage was pulled away by the load and accelerated the loss of hoop function. Theoretically, radial tears result in a loss of hoop function and have been described as functionally equivalent to total meniscectomy [15, 18]. Meniscectomy decreased the contact area and increased (mean, maximum) pressure compared to the intact meniscus. The excision of the meniscus caused the hoop function to collapse, making it impossible to disperse the stress, which is the original function of the meniscus. Therefore, it is possible that the correct load transmission could not be performed through the meniscus, and the load was concentrated on the excised part so that the contact area decreased and the pressure increased. That is, the contact area and the pressure distribution were inversely related to each other due to the excision of the meniscus. These results were similar to those of previous reports and are consistent with reports that meniscectomy leads to an increased risk of developing osteoarthritis [9, 14, 15, 19]. Based on the current study, radial tears should be treated with sutures to obtain the hoop function before the meniscus degeneration in the high-pressure area progresses.

Although rubber sensors are used in several fields, this is the first report to evaluate the biomechanical condition of a meniscal injury model. Additionally, it might have the potential to evaluate the pressure distribution in small animal models because this sensor is highly flexible and easy to customize by changing the substrate size and sensor pitch. This could further become an option for determining meniscal pathophysiology.

The present study had several limitations. First, the pressure distributions were obtained by cutting out only the femur and meniscus to remove various factors and placing the medial meniscus on a planar synthetic bone, as this study is aimed at evaluating the reliability of a novel sensor using porcine meniscus. Future studies should consider a dynamic evaluation of the tibiofemoral joint. Second, this study used a porcine knee. Although the structures of the knees of pigs and humans are similar, the range of motion is different [20], and this might affect biomechanical research.

## 5. Conclusions

The rubber sensor, a novel device for capturing the pressure concentration, is useful for evaluating the pathogenesis and relationship between the pattern of meniscal injury and changes in the biomechanical condition of the knee. The high-pressure area was located around tear, which might deteriorate meniscal injury and weight-bearing cartilage by the loss of load distribution.

## Figures and Tables

**Figure 1:** Novel pressure-sensitive conductive rubber sensor: (a) plane and side view and (b) design drawing (unit: mm).

**Figure 2:** Reliability of the sensor. A compression test was performed using a *φ*10 mm jig in the universal testing machine.

**Figure 3:** (a) Test setup in the universal testing machine to evaluate the contact pressure and area under loads. (b) Representative images of intact, (c) radial tear extending 90%, and (d) partial meniscectomy involving the central 60% of the medial meniscus.

**Figure 4:** Reliability of the sensor: (a) relationship between applied pressure and calculated pressure and (b) color map of pressure distribution.

**Figure 5:** Representative color map of medial meniscal pressure under (a) intact, (b) radial tear extending 90%, and (c) partial meniscectomy involving removal of the central 60%. Calculated results for (d) mean contact pressure, (e) peak contact pressure, and (f) mean contact area.

**Figure 6:** (a) Area analysis results for each pressure region for every 20 N. Areas above 0.4 MPa are indicated by squares. ^∗^*P* < 0.05: radial tear and meniscectomy compared to intact in the area of ≥0.4 MPa. (b) Color map of typical pressure distribution under 20, 60, and 100 N loads.

## Data Availability

The processed data are available from the corresponding author upon request.
